This article has been retracted.

# Liriodenine induces the apoptosis of human laryngocarcinoma cells via the upregulation of p53 expression

**DOI:** 10.3892/ol.2014.2834

**Published:** 2014-12-29

**Authors:** LIANG LI, YING XU, BINQUAN WANG

**Affiliations:** 1 Department of Otolaryngology, Head and Neck Surgery, The Second Affiliated Hospital of Nanjing Medical University, Nanjing, Jiangsu 210011, P.R. China; 2 Department of Otolaryngology, Head and Neck Surgery, The First Hospital, Shanxi Medical University, Taiyuan, Shanxi 030001, P.R. China

**Keywords:** laryngocarcinoma, liriodenine, p53, HEp-2 cells, nude mice

## Abstract

Laryngocarcinoma is one of the most aggressive cancers that affects the head and neck region. The survival rate of patients with laryngocarcinoma is low due to late metastases and the resistance of the disease to chemotherapy and radiotherapy. Liriodenine, an alkaloid extracted from a number of plant species, has demonstrated antitumor effects on multiple types of cancer. However, the effects of liriodenine upon laryngocarcinoma, and the underlying mechanisms, are yet to be elucidated. The present study therefore investigated the potential antitumor effects of liriodenine on HEp-2 human laryngocarcinoma cells *in vitro* and HEp-2-implanted nude mice *in vivo*. Liriodenine induced significant apoptosis and inhibition of cell migration in the HEp-2 cells. Furthermore, the rate of tumor growth in the HEp-2-implanted nude mice was inhibited by the administration of liriodenine. The potential mechanism underlying the antitumor effects of liriodenine may result from an upregulative effect upon p53 expression, which ultimately induces cellular apoptosis. By contrast, the downregulation of p53 significantly reduced the antitumor effects of liriodenine. Together, these results suggest that liriodenine exhibits potent antitumor activities in laryngocarcinoma HEp-2 cells, *in vitro* and *in vivo,* via the upregulation of p53 expression. Liriodenine may therefore be a potential therapy for the treatment of laryngocarcinoma.

## Introduction

Laryngocarcinoma, a cancer of the head and neck region, originates in the squamous cells of the laryngeal epithelium (1), and may develop in any region of the larynx. Smoking, alcohol consumption and other quoted risk factors are reported to be associated with laryngocarcinoma (2). A previous study revealed that in the year 2000, there were 142,000 cases of laryngocarcinoma worldwide (3). Another study estimated a further ~12,500 new cases would arise per year (4). Radiotherapy, chemotherapy and surgery alone, or in combination with therapy, are used for the treatment of laryngocarcinoma. However, during the last 20 years, the five-year post-treatment survival rate has remained poor (2,3). Chemotherapy is an important approach for the treatment of laryngocarcinoma. In comparison with the traditional regimen of surgery followed by radiotherapy, improved organ preservation and survival rates have been demonstrated in patients with chemotherapy-treated laryngocarcinoma (5,6). Therefore, identifying novel, effective chemotherapeutic agents may be essential for the successful treatment of laryngocarcinoma.

Liriodenine is a natural oxoaporphine alkaloid (Fig. 1A) isolated from a number of genera of plant species, including *Fissistigma glaucescens, Annona glabra* and *Liriodendron tulipifera* (7–9). Since 1975, studies have reported on the various biological activities of liriodenine, including its antiplatelet, antimicrobial, antifungal and cardiovascular effects (10–12). *Cyathostemma argenteum* and *Liriodendron tulipifera*, in which liriodenine is the primary effective component, have been shown to exhibit moderate cytotoxic activity against breast cancer and melanoma cell lines (13,14). Therefore, liriodenine has attracted attention for its antitumor activities. A number of studies demonstrated that liriodenine conferred antitumor effects within different tumor cell lines (9,15,16). Furthermore, liriodenine induced DNA damage, reduced the expression of cyclin D1 and cyclin-dependent kinase and decreased the phosphorylation of retinoblastoma protein in tumor cells, which led to G_1_/S phase arrest (17). In addition, the inhibitory effect upon DNA topoisomerase II (18) and the anti-proliferative and apoptosis-inducing actions of liriodenine (15) have been suggested as underlying therapeutic mechanisms. The cytotoxicity of liriodenine may therefore contribute to its antitumor effects. However, the precise mechanism that underlies this action remains to be elucidated.

The aim of the present study was to investigate the antitumor effect of liriodenine on laryngocarcinoma cells in order to evaluate whether it may present a potential antitumor drug for the treatment of laryngocarcinoma.

## Materials and methods

### Reagents

Liriodenine was purchased from ChemBest Research Laboratories, Ltd. (Shanghai, China). All the general reagents used for the cell culture were purchased from Gibco (Carlsbad, CA, USA). Hoechst 33342 and the lectin dyes were purchased from Sigma-Aldrich (St. Louis, MO, USA). The rabbit anti-human monoclonal p53 (1:500 dilution), polyclonal -vascular epidermal growth factor (VEGF; 1:1,000 dilution), polyclonal -cleaved caspase-3 (1:500 dilution) and monoclonal -β-actin (1:5,000 dilution) antibodies were purchased from Cell Signaling Technology, Inc. (Beverly, MA, USA). The rabbit anti-human monoclonal B-cell lymphoma 2 (Bcl-2; 1:500 dilution) and polyclonal -Bcl-2-associated X protein (BAX; 1:500 dilution) antibodies were purchased from Santa Cruz Biotechnology, Inc. (Santa Cruz, CA, USA). Peroxidase-conjugated goat anti-rabbit immunoglobulin G was purchased from Jackson ImmunoResearch Laboratories (West Grove, PA, USA) and the terminal deoxynucleotidyl transferase dUTP nick end labeling (TUNEL) kit was purchased from Roche (Basel, Switzerland).

### Cell culture and transfection

The HEp-2 human laryngeal carcinoma cells were obtained from the American Type Culture Collection (Manassas, VA, USA). The cells were cultured in Dulbecco’s modified Eagle’s medium containing 100 μg/ml penicillin, 100 μg/ml streptomycin and 10% fetal bovine serum (FBS) at 37°C in a humidified CO_2_ incubator, and were subcultured every two to three days. For the following experiments, the cells were trypsinized and harvested upon reaching 70–80% confluency. Adenovirus human *p53* small interfering RNA (Ad-*p53*-siRNA) was obtained from Shanghai Genechem Co., Ltd. (Shanghai, China). The pYr-adshuttle-4 shuttle plasmid, with a titer of 1×10^10^ plaque-forming U/ml, was constructed carrying human *p53* siRNA. A control vector at the same titer was also used in the experiment. The target sequences of the *p53* siRNA and the non-targeting control siRNA were 5′-CCACCAUCCACUACAACUATT-3′ and 5′-UUCUCCGAACGUGUCACGUTT-3′, respectively. Prior to the experiment, the HEp-2 cells were treated with either Ad-*p53*-siRNA or a control vector in an FBS-free culture medium for 16 h, and then incubated with 0.1, 1 or 10 μM liriodenine in a full-culture medium for a further 24 h.

### MTT assay and TUNEL staining

In total, 1×10^4^ HEp-2 cells/well were seeded into 96-well plates and treated with or without adenovirus for 16 h, followed by 0.1, 1 or 10 μM liriodenine for 24 h. The cell viability was then determined using an MTT assay, as previously described (19).

For the TUNEL apoptotic assay, the cells were cultured for 24 h on cover glasses in 12-well plates with 0.1, 1 or 10 μM liriodenine. The apoptotic cells were then detected using the TUNEL commercial kit, according to the manufacturer’s instructions. Images were captured using a DP70 fluorescence microscope (Olympus, Tokyo, Japan). The apoptotic ratio was calculated according to the following equation: Apoptotic ratio = tunnel-positive cells / total cell number.

### Wound healing assay

The HEp-2 cells were added to six-well plates and allowed to reach 90% confluence. Next, the cells were pretreated with 0.1, 1 or 10 μM liriodenine for 2 h, and then scratch wounds were created using a 200-μl pipette tip. The cells were then incubated with the different doses of liriodenine for a further 24 h. The images of the scratched areas were captured at the indicated times with the DP70 microscope (Olympus). The widths of the wounds were measured and the differences calculated.

### Western blot analysis and quantitative polymerase chain reaction (qPCR)

Subsequent to treatment, the cells were lysed using radioimmunoprecipitation assay buffer (Beyotime Institute of Biotechnology, Haimen, China), according to the manufacturer’s instructions. For the *in vivo* experiments, tissues were removed and lysed using radioimmunoprecipitation assay buffer (Beyotime Institute of Biotechnology). The western blot assay, performed as previously described (20), used the cleaved caspase-3, Bcl-2, p53, VEGF and β-actin primary antibodies. The optical density was analyzed with Quantity One software (Bio-Rad Laboratories, Inc., Hercules, CA, USA).

For the qPCR analysis of *p53* expression, the treated HEp-2 cells were lysed using TRIzol (Takara Bio, Inc., Shiga, Japan) in order to isolate the mRNA. The primer oligonucleotides used were synthesized by Biosune Bio (Shanghai, China), and had the following sequences: p53 forward, 5′-TCAACAAGATGTTTTGCCAACTG-3′ and reverse, 5′-ATGTGCTGTGACTGCTTGTAGATG-3′; and β-actin forward, 5′-AATGTCGCGGAGGACTTTGAT-3′ and reverse, 5′-AGGATGGCAAGGGACTTCCTG-3′. The qPCR was performed as previously described (20). Briefly, total RNA (1 μg) was converted to cDNA using M-MLV reverse transcriptase (Takara Bio, Inc.). Next, total RNA was mixed with oligo (dT) at 65°C for 5 min then dNTP was added and samples were incubated at 30°C for 10 min, followed by 60 min at 42°C to collect cDNA. After reverse transcription, the cDNA samples were used to perform qPCR using the SYBR Premix Ex Taq kit (Takara Bio, Inc.) and the Applied Biosystems 7500 Real-Time PCR system (Applied Biosystems, Foster City, CA, USA). The PCR conditions were as follows: 2 min at 50°C, 10 min at 95°C and 40 cycles of 15 sec at 95°C and 1 min at 60°C. The results were expressed as Ct to calculate the relative expression of each mRNA.

### Animal models

Cell suspensions that contained 1×10^8^ cells/ml of normal HEp-2 human laryngeal carcinoma cells or Ad-*p53*-siRNA-pretreated HEp-2 cells were prepared. In total, 0.1 ml of the normal HEp-2 cell suspension was subcutaneously injected into the right upper flank of six-week-old, female, nude BALB/c mice, weighing 20–22 g. When the tumor mass was established at a diameter of ~50 mm, the mice were intraperitoneally injected twice daily with either vehicle (10 ml/kg saline) or 50 mg/kg liriodenine. In the *p53*-siRNA-treated group, the mice were implanted with Ad-*p53*-siRNA-pretreated HEp-2 cells, and then injected with vehicle (not effective on tumor growth; data not shown) or liriodenine for 15 consecutive days, according to the same schedule as the normal HEp-2 cell-implanted mice. The behavior of the animals was observed daily, and tumor measurements were recorded every two days. The short (r) and long (l) diameters of the tumors were measured, and the tumor volume of each was calculated according to the following equation: Tumor volume = (r × l) / 2. Following 15 days of drug administration, the mice were sacrificed by CO_2_ inhalation, and the sizes and weights of the tumors were recorded and then the tumors treated for continuous experiments. The animal studies were permitted and carried out according to the guidelines for animal experiments, as outlined by the Committee for Animal Experiments of the First Hospital, Shanxi Medical University (Taiyuan, China).

### Immunohistochemistry

The subcutaneous tumors removed from the mice were cut and processed for immunostaining, as previously described (21). The tumor tissues were then frozen in OCT, and 10-μm frozen sections were prepared. Subsequent to air-drying for 30 min, the sections were fixed in cold acetone and washed with phosphate-buffered saline (PBS). Next, hematoxylin and eosin (HE) staining was performed in order to observe the morphology of the tumor tissues. The TUNEL assay was performed in order to detect the apoptotic cells within the tumor tissues, according to the manufacturer’s instructions. Lectin staining was performed to mark the blood vessels and evaluate the extent of angiogenesis within the tumor tissues. The specimens were incubated with 3% H_2_O_2_ in methanol for 15 min at room temperature to block endogenous peroxidase, and then incubated for 20 min at room temperature in PBS containing 1% bovine serum albumin for protein blocking. The lectin staining was then performed. All images were captured using a DP70 fluorescence microscope (Olympus).

### Statistical analysis

Statistical data are expressed as the mean ± standard error. The differences between groups were analyzed using a two-sided t-test, an analysis of variance and Dunnett’s test. P<0.05 was used to indicate a statistically significant difference.

## Results

### Liriodenine induces apoptosis and the inhibition of cell migration in HEp-2 cells

In order to investigate the antitumor effects of liriodenine in the human laryngeal carcinoma HEp-2 cell line, an MTT assay was performed to analyze the cellular viability. Following a 24-h treatment, liriodenine induced a dose-dependent decrease in the cellular viability of the HEp-2 cells, with a half maximal inhibitory concentration (IC_50_) of 2.332 μM (Fig. 1B). The present study then investigated whether the observed liriodenine-induced decrease in cell viability was a result of apoptosis. TUNEL staining was performed to determine the apoptotic rate of liriodenine-treated HEp-2 cells. Following a 24-h incubation with liriodenine, the samples contained fewer living cells and more TUNEL-positive nuclei, exhibited in a dose-dependent manner (Fig. 1C and D). In addition, certain apoptotic biomarkers were investigated by western blot analysis. Within the HEp-2 cells, liriodenine reduced the expression of Bcl-2, and increased the expression of p53 and cleaved caspase-3 in a dose-dependent manner (Fig. 1E).

Furthermore, in order to detect whether liriodenine affected cellular migration, a wound-healing assay was performed upon the HEp-2 cells. As shown in Fig. 1F and G, 1 μM liriodenine significantly suppressed cellular migration compared with the control. Together, the results indicated that liriodenine induced the apoptosis and migration of the HEp-2 cells with a high efficacy. This suggested that liriodenine may be a potential anti-laryngocarcinoma compound.

### Downregulation of p53 expression suppresses the pro-apoptotic effect of liriodenine

The protein, p53, possesses a key role in tumor growth (22). In response to cellular stresses, p53 induces cell cycle arrest and apoptosis via a DNA damage response (23). Similar to the results reported by Hsieh *et al* (9), the present study demonstrated that liriodenine could dose-dependently increase p53 expression in the HEp-2 cells (Fig. 1E). Using flow cytometry, Hsieh *et al* (9) identified that treatment with liriodenine increased the number of p53-positive cells (9). The present study confirmed that 10 μM liriodenine increased p53 expression in a time-dependent manner (Fig. 2A and B). In order to further investigate the role of p53 in liriodenine-mediated tumor inhibition, an adenoviral vector, containing human *p53* siRNA, was used to knock down *p53* expression. The expression of *p53* mRNA was significantly reduced in the siRNA-treated HEp-2 cells (Fig. 2C). Furthermore, the liriodenine-induced increase in *p53* mRNA expression was reversed by the *p53*-siRNA (Fig. 2C). A similar pattern was observed for p53 protein expression (Fig. 2D and E). Consequently, there was a >6-fold increase in the IC_50_ of liriodenine in the *p53*-siRNA-treated HEp-2 cells (15.68 vs. 2.332 μM; Fig. 2F). The liriodenine-induced elevation in the expression of cleaved caspase-3 was almost abolished in the *p53*-siRNA-treated HEp-2 cells (Fig. 2D and G). Together, these data indicated that p53 plays an important role in the mechanism of liriodenine-induced apoptosis in the HEp-2 cells.

### Liriodenine attenuates the rate of tumor growth in HEp-2-transplanted nude mice via upregulating the expression of p53

The HEp-2-transplanted nude mice were utilized for the efficacy studies as previously described (24). Subsequent to cell transplantation, the administration of liriodenine was initiated when the size of the tumors had reached 0.05 cm^3^. Following 15 days of treatment, no significant change in body weight and food intake was identified between each group (data not shown). Treatment of the mice with 50 mg/kg body weight liriodenine inhibited the growth of the tumors that had originated from the HEp-2 human laryngeal carcinoma cells (Fig. 3A). However, the antitumor effect of liriodenine in the animals implanted with Ad-*p53*-siRNA-pretreated HEp-2 cells was notably suppressed (Fig. 3A). At the end of the treatment period, the tumor tissues were removed and weighed. The therapeutic effect of 50 mg/kg liriodenine in the mice injected with Ad-*p53*-siRNA-pretreated HEp-2 cells was markedly less compared with that observed in normal HEp-2 cell-injected mice (Fig. 3B).

To further investigate the effect of *p53*-siRNA upon the antitumor effects of liriodenine *in vivo*, a morphological study was performed. Upon HE staining, the tumor tissue sections from the liriodenine-treated group demonstrated extensive necrosis (Fig. 3C). Therefore, apoptotic cells were further analyzed using TUNEL staining. Overall, there were more TUNEL-positive nuclei visible in the liriodenine-treated groups compared with the vehicle group (Fig. 3C). The expression of cleaved caspase-3 within the tumor tissues was also increased following treatment with liriodenine (Fig. 3D). However, the liriodenine-treated mice injected with *p53*-siRNA HEp-2 cells demonstrated fewer apoptotic cells and lower expression of cleaved caspase-3 compared with the mice that received 50 mg/kg liriodenine alone (Fig. 3C and D). The liriodenine-induced upregulation of p53 in the transplanted tumor tissues was inhibited in the *p53*-siRNA group (Fig. 3D), which indicated that liriodenine-induced apoptosis may function through the p53 pathway.

Although the cells preconditioned with *p53*-siRNA demonstrated a reduced response to liriodenine in the HEp-2-transplanted mice, the suppressive effect upon liriodenine-induced apoptosis was not as notable as that observed in the *in vitro* experiment. Therefore, the antitumor mechanism of liriodenine *in vivo* was further studied. Angiogenesis is another important factor known to accelerate tumor growth (25). Therefore, to confirm whether the antitumor effect of liriodenine *in vivo* was associated with angiogenesis, lectin dye was used to mark blood vessels within the tumor tissues. Overall, no significant reduction in the number of lectin-positive cells was observed in the groups treated with *p53*-siRNA and liriodenine, or with liriodenine alone (Fig. 3C). In addition, western blot analysis was used to confirm the expression of VEGF, a factor associated with tumor angiogenesis (26). In accordance with the unchanged vessel density within the tumor tissues, there was no evident change in the expression of VEGF in each group (Fig. 3D). Taken together, the present study results concluded that cytotoxicity, but not angiogenesis, was associated with the *in vivo* antitumor effects of liriodenine, and that p53 expression had a crucial role in this process.

## Discussion

Liriodenine has been proposed as a tumor inhibitor since 1969 (7). However, as a potential antitumor drug, the pharmacological activity and underlying therapeutic mechanisms of liriodenine are yet to be elucidated. The present study demonstrated that increased apoptosis and inhibition of cellular migration could be induced by liriodenine in HEp-2 cells. Furthermore, the *in vivo* study provided evidence that liriodenine may be a potential antitumor compound with limited toxicity. In addition, by using a *p53*-siRNA-expressing adenovirus vector, the present study identified the crucial role of p53 in liriodenine-induced tumor inhibition, *in vitro* and *in vivo*.

It is widely known that p53 acts as tumor suppressor in human carcinomas via the regulation of the cell cycle and cellular apoptosis (27). A number of studies have confirmed that p53 expression is associated with chemotherapeutic agent-induced inhibition of tumor growth in multiple cancers, including laryngocarcinoma (28,29). During tumor growth, p53 can be activated by cytotoxic stressors (30) to induce cell cycle arrest, DNA damage and cellular apoptosis (31). Therefore, the targeting of p53 regulatory pathways has been considered during the development of antitumor drugs. Several compounds with potent antitumor activity have already been revealed to be associated with p53 regulation (28,29). Furthermore, *p53*-expressing adenoviruses have also been proven to confer antitumor effects in clinical tests (32). Therefore, the combination of p53-based therapies with other current therapies may be effective for the treatment of tumors, including laryngocarcinoma (33). A previous study reported that liriodenine increased the number of p53-positive cells in human hepatoma cells (9). Therefore, the effect of liriodenine on HEp-2 cells may be associated with p53 expression. The present study confirmed that liriodenine induced a significant increase in the expression of p53 in a dose- and time-dependent manner. Furthermore, liriodenine also reduced the level of the key anti-apoptotic protein, Bcl-2, which may be due to p53-mediated negative regulation (34). This process finally activated caspase-3, and contributed to cellular apoptosis. Using an adenovirus vector, it was revealed that the downregulation of p53 notably suppressed the antitumor effects of liriodenine, *in vitro* and *in vivo*. Therefore, p53 expression could play a crucial role in liriodenine-induced cytotoxicity within laryngocarcinoma HEp-2 cells.

The *in vivo* inhibitory effect of *p53*-siRNA upon liriodenine-induced apoptosis was not as effective as that observed in the *in vitro* experiment. In addition, the effect of liriodenine upon the extent of angiogenesis was investigated using a xenograft. Unexpectedly, there was no observable change in angiogenesis following treatment with liriodenine. Therefore, in addition to the upregulation of p53 expression, but excluding the inhibition of angiogenesis, there may be other anti-tumor mechanisms contributing to liriodenine-induced tumor cell apoptosis *in vivo*. Tumor necrosis and inflammatory-related pathways may also be associated with the antitumor activity of liriodenine. The duration of the effect of Ad-*p53*-siRNA may also contribute to the differences observed between *in vivo* and *in vitro* experiments. Further studies are therefore required to examine the detailed pharmacological mechanisms that underlie the action of liriodenine.

In conclusion, the present study demonstrated that liriodenine conferred potent antitumor activities in laryngocarcinoma HEp-2 cells, *in vitro* and *in vivo*. The potential mechanism underlying the antitumor effects of liriodenine may result from an upregulatory effect upon p53 expression, which ultimately induces cellular apoptosis. It is therefore suggested that liriodenine may be a potential therapy for the treatment of laryngocarcinoma.

## Figures and Tables

**Figure 1:** Liriodenine administration induces apoptosis and the inhibition of cellular migration in HEp-2 cells. (A) The structure of liriodenine, 8H-benzo[g]-1,3-benzodioxolo[6,5,4-de]-quinolin-8-one. (B) IC_50_ non-linear fit curve showing the effect of varying concentrations of liriodenine on the cellular viability of HEp-2 cells, which was determined by MTT assay. (C) Terminal deoxynucleotidyl transferase dUTP nick end labeling (TUNEL) revealing apoptotic cells. TUNEL-positive cells were identified by green fluorescence. All nuclei were stained blue with Hoechst 33342. Scale bar referring to all panels, 100 μm. (D) The cellular apoptotic rate according to the different concentrations of liriodenine was calculated. ^*^P<0.05 and ^***^P<0.001 compared with the vehicle-treated group (n=10). (E) Western blot analysis revealing the expression of B-cell lymphoma 2 protein (Bcl-2), p53 and cleaved caspase-3 following treatment with different concentrations of liriodenine. β-actin was used as the internal control. All blots were repeated at least three times. (F) Effect of 1 μM liriodenine upon cellular migration was investigated. Representative images revealing the extent of migration at specific time-points following treatment. Scale bar referring to all panels, 10 μm. (G) Wound width was measured and the relative values are presented. ^**^P<0.01 and ^***^P<0.001 compared with the vehicle-treated group (n=3). IC_50_, half maximal inhibitory concentration.

**Figure 2:** Downregulation of p53 expression suppresses the pro-apoptotic effect of liriodenine. (A) Western blot analysis revealing the expression of p53 at different times following treatment with 10 μM liriodenine. β-actin was used as the internal control. Blots were repeated at least three times for statistical analysis. (B) Statistical analysis of p53 expression at different times following treatment with 10 μm liriodenine. ^**^P<0.01 and ^***^P<0.001 compared with the vehicle-treated group (n=3). (C) Expression of p53 mRNA, following treatment with liriodenine in the presence or absence of p53-small interfering RNA (siRNA), was determined by quantitative polymerase chain reaction. ^***^P<0.001 compared with the vehicle-treated group (n=3). (D) Western blot analysis revealing the expression of p53 and cleaved caspase-3 following treatment with liriodenine. β-actin was used as the internal control. Blots were repeated at least three times for statistical analysis. Statistical analysis of (E) p53 and (F) cleaved caspase-3 expression following treatment with liriodenine, in the presence or absence of p53-siRNA. ^**^P<0.01 and ^***^P<0.001 compared with the vehicle-treated group. (G) The effect of liriodenine upon the cellular viability of p53-siRNA-infected HEp-2 cells was determined by MTT assay.

**Figure 3:** Liriodenine attenuates the rate of tumor growth in HEp-2-transplanted nude mice via the upregulation of p53 expression. (A) Tumor volume was measured every two days and calculated according to the formula described in the Materials and methods section. ^*^P<0.05 and ^***^P<0.001 in liriodenine alone-treated group compared with the vehicle-treated group (n=8). ^#^P<0.05 in the liriodenine-p53-small interfering RNA (siRNA)-treated group compared with the vehicle-treated group (n=8). (B) Macroscopic appearance of tumor tissues removed from each group. Scale bar referring to all panels, 1 cm. (C) Morphological analysis of tumor tissues. Following treatment, tumor tissues from vehicle-, liriodenine- and liriodenine-p53-siRNA-treated nude mice were removed and sectioned. Hematoxylin and eosin staining revealing blue-stained nuclei and pink-stained cytoplasm. Green fluorescence revealing lectin-positive vessels. Brown nuclei revealing TUNEL-positive cells. Representative scale bars are indicated for each panel. (D) Western blot analysis revealing the expression level of vascular epidermal growth factor (VEGF), p53 and cleaved caspase-3 in the tumor tissues following treatment. β-actin was used as the internal control. Each blot was repeated three times from tissues obtained from different mice. TUNEL, terminal deoxynucleotidyl transferase dUTP nick end labeling.
